# Effects of “Mindfulness Acceptance Insight Commitment” Training on Flow State and Mental Health of College Swimmers: A Randomized Controlled Experimental Study

This article has been retracted.

**DOI:** 10.3389/fpsyg.2022.799103

**Published:** 2022-06-24

**Authors:** Jun-hui Ning, Qing-wei Hao, Da-cai Huang

**Affiliations:** School of Martial Arts and Dance, Shenyang Sport University, Shenyang, China

**Keywords:** mindfulness training, college swimmers, flow state, mental health, randomized controlled trial

## Abstract

This research explores the intervention effect of the mindfulness acceptance insight commitment (MAIC) training program on the mindfulness level, flow state, and mental health of college swimmers. A sample of 47 college swimmers from a regular university was recruited and randomly divided into two groups before the intervention. Independent variables between groups are psychological training mode (MAIC training/no training), and the independent variable within group was time (pre-test, post-test, and continuity test). The dependent variables are mindfulness level, flow state, and mental health (anxiety, depression, training, and competition satisfaction). Results show that after the intervention of MAIC training, the mindfulness level of athletes’ flow state has been significantly improved, whereas anxiety and depression significantly decreased. In addition, the satisfaction with training and competition significantly improved. In the continuous stage after the intervention, the mindfulness level, flow state, and mental health of athletes are still significantly higher than those in the pre-test. The comparison of the post-test and continuity test show no significant differences in the mindfulness level, flow state, depression, and training and competition satisfaction of athletes. Still, the anxiety level shows an upward trend with a significant difference. This study demonstrates that the MAIC mindfulness training program can significantly improve the mindfulness level, flow state, anxiety, depression, and training and competition satisfaction of college swimmers with a good continuity effect. Thus, the athletes’ sports experience can be improved, and good psychological benefits can be attained.

## Introduction

College athletes, as both students and athletes, can be considered a special group (Xian-ming and Dong-lin, 2007). A general belief is that college is a relaxing time, but with the increasing pressure of social competition, college athletes face the combined pressures of academic tasks, sports training and competition, and the emergence of sports time limits and injury (Reardon et al., 2019). These athletes are prone to emotional management and pressure control problems, which lead to a high prevalence of mental disorders, such as anxiety, depression, pain, and eating concerns. The two-factor model of mental health assumes two dimensions: positive and negative mental states (Keyes, 2012). In terms of positive psychological state, training and competition satisfaction have been shown as an important index that can predict athletes’ pre-competition emotion and is significantly negatively correlated with their psychological fatigue (Lundqvist and Sandin, 2014). In addition, anxiety and depression are common negative psychological states among athletes (Rice et al., 2016). These mental health problems potentially affect their sports performance (Jain and Thomas, 2002; Hanton et al., 2005).

Impact of mental health on flow state. In the field of sports psychology, a flow state is defined as “an optimal experience state, that is, the state of consciousness in which athletes are committed to focusing on their tasks and creating the best sports performance” (Swann et al., 2018). When athletes devote themselves to their activities, they can create a “catalyst” to experience a flow state, resulting in immersion and loss of self. Considering the importance of a positive mental state to sports performance, heart flow has an increasing potential to improve athletes’ sports performance (Jackson et al., 2001; Rhodes and Andrew, 2015). In the flow state, the athlete and the environment are harmonious, which is manifested in the automatic control of movement. In essence, this is an optimal psychological state. With the flow state, the athlete can effectively prevent or offset disharmonious relationships with the environment to enable excellent performance, becoming the basis for athletes to achieve exceptional sports results (Wei-na and Liu, 2009; Latinjak and Hatzigeorgiadis, 2021). However, the flow state of athletes can be affected by cognitive, emotional, mental health, and other factors, which also affect the feeling of athletes in the competition and flow state. When athletes experience anxiety, depression, and other emotions in the preparation or competition, a negative concentration of self-consciousness occurs. As such, athletes cannot feel the flow state, which affects their sports performance (Chen et al., 2018).

Effect of mindfulness training on flow state and mental health. Mindfulness training is a psychological and behavioral training method based on acceptance. The belief is that excellent behavior can still be achieved even when accompanied by a negative psychological state. Such training advocates for detecting and accepting internal psychological events without judgment. At the same time, internal psychological events are decentralized to shift the focus of attention from the self to the task and devote itself to the current behavioral process. Mindfulness training has shown its effectiveness in the field of clinical psychology. Widely used to regulate emotions and relieve stress, mindfulness training can improve the level of anxiety and depression of college students (Zhong Jiahan and Bo, 2015; Li et al., 2020). In the field of medicine, mindfulness training has also been proven effective in addressing pain, anxiety, depression, stress, and eating disorders, such as Mindfulness-Based Stress Reduction (MBSE) (Kabat-Zinn, 2015). Moreover, mindfulness training has many similarities with the flow state concept in the field of sports psychology. For example, mindfulness can promote attention regulation, emotion regulation, and body consciousness by focusing on the current task. Kee and Wang (2012) found that the higher the mindfulness trait of athletes, the higher their flow state scores in challenging skill balance, clear goal, attention concentration, and sense of control. Acceptance-based intervention methods are used to improve the performance level of athletes, which confirms the effectiveness of enhancing their flow state experience in the field of sports (Kabat-Zinn et al., 1985; Kaufman et al., 2009; Schwanhausser, 2009; Hasker, 2010).

“Mindfulness acceptance insight commitment” (MAIC) training. The mindfulness training methods developed by western scholars have received much empirical research but may be “acclimatized” when directly used for Chinese athletes. Therefore, Gangyan (2014) introduced “consciousness” in Zen thoughts on the basis of traditional mindfulness training and in combination with China’s local social and cultural conditions, and thus developed the MAIC training. This program is an acceptance-based psychological and behavioral training method, which integrates the adversity coping theory of local scholars, oriental Zen thoughts, and the skills of third-generation cognitive behavioral therapy. As an attempt by Chinese scholars to develop a mindfulness training system based on local culture and practices (Gangyan et al., 2014), the MAIC training program extracts three skills from Zen thoughts, namely “mindfulness,” “decentralization,” and “acceptance.” The aim is to help athletes better perceive and invest in the current behavior process, that is, to treat the current behavior tasks with a mindfulness attitude rather than to judge or respond to inner experiences—especially negative ones—and accept their existence calmly. The focus of attention must shift from the self-concern of eliminating or controlling the internal experience to the task of behavior performance and fully participating in the present behavioral process (Weirui and Lu, 2010). The MAIC training program also cites the “values” and “input” in the western third-generation cognitive behavioral therapy to provide direction for current behavior, promote the connection between values and specific behavior, and realize the long-term adherence to values. In addition, through the improvement of Zen thoughts—consciousness, individual values can be adjusted. The MAIC training program includes seven parts of mindfulness training content, which pays attention to the operability of the implementation, from the most basic practice to daily application in life and then to special projects. MAIC training is expected to become a psychological intervention that can improve the mental health level of athletes and their sports performance. However, at present, MAIC training research is only limited to several elite athletes, most of whom are under case studies (Danran and Gangyan, 2014). Considering the problems of mental health and sports performance faced by college athletes, the introduction of more effective psychological training methods is necessary.

Based on the above discussion, this study explores the effects of MAIC training on the mindfulness level, flow state, and mental health of college swimmers. According to such purpose, this study proposes two hypotheses: (1) compared with the control group, the mindfulness level, flow state, and mental health of college athletes trained by MAIC are significantly improved; (2) after MAIC training intervention, the athletes gain better continuity effect of flow state and mental health.

## Materials and Methods

### Experimental Participants

College athletes refer to the students who are officially admitted by colleges and universities with the title of national athletes at or above level 2 according to China’s enrollment policy for high-level athletes every year. Based on the actual situation of colleges and universities, the high-level college athletes in this study refer to the college students who have obtained the national second-class athlete certificate (included) or equivalent to the national second-class athlete level and participate in the regular training of the school team and complete the school competition task. A total of 47 college swimmers (23 women) were recruited for the intervention experiment. The participants were 19–25 years old (average age: 22.34 years; SD: 2.17). All participants had more than 5 years of swimming experience, and the swimming time per week was more than 20 h. All 47 (100%) athletes completed the seminar. Before the experimental intervention, all athletes said they had no experience with psychological skills training intervention and no history of neurological diseases or cognitive impairment in daily life.

### Experimental Measurement Tools

#### Five Facet Mindfulness Questionnaire

The scale was developed by Baer et al. (2006), to measure the level of mindfulness ability of individuals. The questionnaire contains 39 questions, including observation, description, conscious activity, non-judgment, and non-reaction. In the Likert 5-point scoring system, the higher the total score from “1” (totally disagree) to “5” (totally agree), the higher the individual mindfulness ability. The consistency coefficient of Five Facet Mindfulness Questionnaire (FFMQ) was 0.746.

#### Short Flow State Scale

The scale was revised by Wei-na (2010) of East China Normal University. Short Flow State Scale (SFSS) was used to evaluate the flow state immediately after the end of the activity. The scale has nine questions on nine dimensions of flow state: challenge skill balance, action awareness, clear goal, clear feedback, focusing on the task at hand, sense of control, loss of self-awareness, time conversion, and enjoyable experience. In the Likert 5-point scoring system, the higher the total score from “1” (totally disagree) to “5” (totally agree), the higher the individual flow state. The consistency coefficient of SFSS was 0.73.

#### Competitive State Anxiety Inventory-2

Revised by Beili (1993), this scale has 27 items, including cognitive state anxiety, physical state anxiety, and state self-confidence. A 4-point Likert scoring system was adopted. From “1” (not at all) to “4” (very strong), the higher the score, the higher the athlete’s anxiety level. The consistency coefficient of Competitive State Anxiety Inventory-2 (CSAI-2) was 0.72.

#### Profile of Mood State

The scale was revised by Beili (1995). Profile of Mood State (POMS) was used to evaluate the mood state of athletes. The questionnaire includes seven dimensions: tension, anger, fatigue, depression, energy, panic, and self. Given that this study only discusses depression, only the results of the depression dimension are selected for data analysis. A 4-point Likert scoring system from “0” (almost none) to “4” (very) is adopted, the higher the score, the higher the level of depression of athletes. The internal consistency reliability of the scale was 0.71, which can better reflect individual emotional status.

#### Training and Competition Satisfaction Questionnaire

The scale was designed by Liwei and Zhanpeng (2002). Training and Competition Satisfaction Questionnaire (TCSQ) is used to evaluate athletes’ training and competition satisfaction. The scale has six questions scored on a 7-point Likert system from “1” (absolutely incorrect) to “7” (always correct). The higher the score, the higher the athlete’s training and competition satisfaction. The internal consistency reliability of the scale was 0.75.

### Experimental Design

This study used a randomized controlled experimental RCT design on a single-blind test. As shown in Figure 1. Before the intervention, all subjects were randomly divided into two groups, 24 in the MAIC training group (11 females) and 23 in the control group (12 females). The independent variables between groups were psychological training modes (MAIC training/no training) and within the group were time-related: pre-test (T1), post-test (T2), and continuity test (T3), that is, 10 weeks after the end of the intervention. The dependent variables were mindfulness level, flow state, and mental health (anxiety, depression, training, and competition satisfaction).

**FIGURE 1:** Experimental steps.

### Mindfulness Acceptance Insight Commitment Curriculum

The athletes in the MAIC group received training intervention once a week for 7 weeks (Table 1). Each session lasted for 60–90 min. After the intervention, the athletes were followed up for 10 weeks. The training was supplemented with a mindfulness intervention log as supervision and guidance. The content was planned to be designed with reference to the mindfulness training manual for professional athletes (Gangyan, 2014). The training was carried out in a quiet and comfortable room operated by scholars majoring in applied psychology with mindfulness training experience to avoid interference. A payment was offered to the participants to ensure that they could seriously and carefully accept the MAIC training intervention. The control group did not receive any intervention. All psychological variables were evaluated three times: pre-test (T1), post-test (T2), and continuity test (T3).

**TABLE 1:** Mindfulness acceptance insight commitment course arrangement.

Course theme	Course content	Practice
1. Mindfulness training preparation	Introduce the basic concept, key points, and functions of “mindfulness acceptance insight commitment”; introduce intervention methods	Centering exercise
2. Mindfulness training guidance	Introduce the concept of “mindfulness”; analyze the relationship between mindfulness and behavior	Mindfulness breathing practice, internal observation practice
3. Decentralization	Introduce the concept of “decentralization”	Mindfulness walking practice, number practice
4. Acceptance	Introduce the concept of “acceptance”; analyze the relationship between “experience acceptance and avoidance” and sports performance	Mindfulness yoga practice
5. Values and awareness	Introduce the concept of “values and insight”; explain the relationship between values and insight	Mindfulness meditation, body scanning
6. Investment	Introduce the concept of “commitment and concentration”	Selfless behavior practice
7. Review	Review the basic concept of “mindfulness acceptance insight commitment”; review mindfulness training; emphasize the importance of mindfulness training	Comprehensive practice

### Statistical Method

In this study, the repeated measurement ANOVA method was used to analyze and test the inter- and intra-group variables and the data met homogeneity of variance and spherical symmetry before analysis. Among the data, the intervention type (MAIC group and control group) was used as the inter-group variable, the measurement time (T1, T2, T3) was used as the intra-group variable, and the mindfulness level, flow state, and mental health (anxiety, depression, and satisfaction with training and competition) were measured as dependent variables. ANOVA was followed by further *post hoc* multiple comparisons. An independent sample *t*-test was used to test the difference between groups, and paired sample *t*-test was used to test the difference in variation within groups. The baseline scores are shown in Table 2.

**TABLE 2:** Baseline scores.

	MAIC group			Control group		
	*N*	*M*	SD	*N*	*M*	SD
**Mindfulness**						
Pre-test	24	119.25	12.052	23	118.78	12.674
Post-test	24	134	16.759	23	118.65	12.452
Continuity test	24	133.54	16.352	23	118.91	12.083
**Flow state**						
Pre-test	24	29.5	1.642	23	29.43	1.647
Post-test	24	33.13	0.992	23	29.22	1.833
Continuity test	24	33.87	1.191	23	29.91	2.661
**Anxiety**						
Pre-test	24	58.5	1.142	23	58.43	1.121
Post-test	24	52.08	1.717	23	58.39	1.118
Continuity test	24	53.83	1.926	23	58.87	1.456
**Depressed**						
Pre-test	24	3.25	0.737	23	3.22	0.736
Post-test	24	2.29	0.464	23	3.13	0.694
Continuity test	24	2.42	0.584	23	3.3	0.822
**Training and competition satisfaction**						
Pre-test	24	22.46	1.103	23	22.43	1.121
Post-test	24	26.17	1.685	23	22.39	1.118
Continuity test	24	25.92	1.613	23	22.48	0.947

## Results

### Effect of Mindfulness Acceptance Insight Commitment Training on the Mindfulness Level of College Swimmers

Figure 2 shows the results of mindfulness level scores in the MAIC and control groups. Repeated measurement ANOVA shows that the mindfulness levels of the two groups, “Group” × “Time” interaction is significant [*F*(2,90) = 90.922, *p* < 0.001, η_p_^2^ = 0.644].

**FIGURE 2:** Comparison of mindfulness scores between the MAIC and control groups.

#### Comparison of Real-Time Test Results of Mindfulness Level

Through MAIC training intervention, the comparison of the pre-test and post-test in the MAIC group shows a significant difference, and the post-test effect is better than the pre-test effect (MD = 14.750, *p* < 0.001). No significant difference is observed between the pre-test and post-test in the control group (MD = −0.130, *p* = 0.999). In the post-test comparison between the MAIC and control groups, the mindfulness level of the MAIC group is significantly higher (MD = 15.348, *p* = 0.001). The above results show that MAIC training improves the mindfulness level of participants.

#### Comparison of the Effect of Mindfulness Level Continuity Test

In the MAIC group, the comparison of the pre-test and continuity tests shows a significant difference. The effect of the continuity test is better than that of the pre-test (MD = 14.292, *p* < 0.001) but not significantly different from the post-test (MD = −0.458, *p* = 0.595). In the control group, no significant difference is observed between the pre-test and continuity test (MD = 0.130, *p* = 0.999) or between the post-test and continuity test (MD = −0.261, *p* = 0.895). In comparing the continuity test between the MAIC and control groups, the mindfulness level of the MAIC group is significantly higher (MD = 14.629, *p* = 0.001). The above results show that the continuous effect of MAIC intervention is better, and thus continuous training may be more beneficial to improving mindfulness.

### Effect of Mindfulness Acceptance Insight Commitment Training on the Flow State of College Swimmers

Figure 3 shows the flow state scores in the MAIC and control groups. Repeated measurement ANOVA shows that the flow state of the two groups “Group” × “Time” interaction is significant [*F*(2,90) = 46.629, *p* < 0.001, η_p_^2^ = 0.509].

**FIGURE 3:** Comparison of flow state scores between MAIC group and control group.

#### Comparison of Flow State Real-Time Test Results

Through MAIC training intervention, the comparison of pre-test and post-test in the MAIC group shows a significant difference, and the post-test effect is better than the pre-test effect (MD = 3.625, *p* < 0.001). No significant difference is observed between the pre-test and post-test in the control group (MD = 0.217, *p* = 0.841). The flow state level of the MAIC group is significantly higher than that of the control group (MD = 3.908, *p* < 0.001). The above results show that MAIC training improves the flow state of participants.

#### Comparison of Flow State Continuity Test Results

In the MAIC group, a comparison of the pre-test and continuity test shows a significant difference. The effect of the continuity test is better than that of the pre-test (MD = 4.375, *p* < 0.001). No significant difference is observed in the comparison of post-test and continuity test (MD = −0.750, *p* = 0.138). In the control group, no significant difference is observed between the pre-test and continuity test (MD = −0.478, *p* = 0.606) and between the post-test and continuity test (MD = −0.696, *p* = 0.200). In the comparison of the continuity test between the MAIC group and the control group, the flow state of the MAIC group is significantly higher than that of the control group (MD = 3.962, *p* < 0.001). The above results show that the training continuity effect of the MAIC group is better and reflects the importance of spontaneous MAIC training to improve the flow state of athletes.

### Effect of Mindfulness Acceptance Insight Commitment Training on the Mental Health of College Swimmers

Figure 4 shows the results of mental health levels in the MAIC and control groups. The repeated measurement ANOVA shows that “Group” of training and competition satisfaction level × “Time” interaction is significant [*F*(2,90) = 70.733, *p* < 0.001, η_p_^2^ = 0.611]; “Group” of anxiety level × “Time” interaction is significant [*F*(2,90) = 159.618, *p* < 0.001, η_p_^2^ = 0.770]; “Group” of depression × “Time” interaction is significant [*F*(2,90) = 19.378, *p* < 0.001, η_p_^2^ = 0.301].

**FIGURE 4:** Comparisonof mental health scores between the MAIC group and control group. **(A)** Comparison of training and Competition Satisfaction between MAIC group and control group. **(B)** Comparison of depression between MAIC group and control group. **(C)** Comparison of anxiety between MAIC group and control group.

#### Comparison of the Effects of Immediate Mental Health Testing

Through MAIC training intervention, significant differences are observed in the pre-test and post-test of anxiety, depression, training, and competition satisfaction in the MAIC group. The post-test effect is better than the pre-test effect (MD = 6.417, *p* < 0.001), (MD = 0.958, *p* < 0.001), and (MD = 3.708, *p* < 0.001). No significant difference is observed between the pre-test and post-test in the control group (MD = 0.043, *p* = 0.998), (MD = 0.087, *p* = 0.783), and (MD = 0.043, *p* = 0.998). In the post-test comparison between the MAIC and control groups, the three indexes of anxiety, depression, and training and competition satisfaction in the MAIC group are significantly better than those in the control group (MD = −6.308, *p* < 0.001), (MD = −0.839, *p* < 0.001), and (MD = 3.775, *p* < 0.001). The above results show that MAIC training can reduce the anxiety and depression level of athletes and improve the satisfaction of athletes in training and competition.

#### Comparison of Continuity Test Results of Mental Health

In the MAIC group, comparison of the pre-test and continuity test of anxiety, depression, and training and competition satisfaction show significant differences. The effect of the continuity test is better than that of the pre-test (MD = −4.667, *p* < 0.001), (MD = −0.833, *p* < 0.001), and (MD = 3.292, *p* < 0.001). However, the comparison of the post-test and continuity test shows no significant difference in the depression level and training and competition satisfaction in the MAIC group (MD = −0.125, *p* = 0.622), (MD = −0.250, *p* = 0.102) but has a significant difference in anxiety level compared with the post-test (MD = −1.750, *p* < 0.001). In the control group, no significant difference is observed in the effects of the pre-test and continuity tests of the three indexes (MD = −0.44, *p* = 0.780), (MD = 0.087, *p* = 0.783), and (MD = −0.43, *p* = 0.998) or in the post-test and continuity test (MD = −0.478, *p* = 0.057), (MD = −0.174, *p* = 0.366), and (MD = −0.087, *p* = 0.846). In the comparison of the continuity test between the MAIC and control groups, the anxiety, depression, and training and competition satisfaction indexes of the MAIC group are significantly better than those of the Control group (MD = −5.036, *p* < 0.001), (MD = −0.888, *p* < 0.001), and (MD = 3.438, *p* < 0.001). The above results show that mindfulness training has a good continuous effect on improving athletes’ anxiety, depression, and training and competition satisfaction. However, after the end of the MAIC intervention, athletes’ anxiety and depression levels have increased while training and competition satisfaction has decreased.

## Discussion

Through experiments, this study verifies the effect of the MAIC mindfulness training method based on the local design on the flow state and mental health of college athletes. The scores of the five-factor mindfulness scale show that the intervention of MAIC training has significantly improved the mindfulness level of athletes, which in turn helps them better perceive their own sports conditions and actively deal with the negative emotions in daily life, and thus focus on the current task and improve their sports performance. Mindfulness training can improve athletes’ mindfulness ability (Guoyan and Gangyan, 2015; Danran and Zhe, 2016), which is also considered one of the ways to improve sports performance. The present study confirms this view. In terms of the pre-test and continuity test, the mindfulness level of athletes is maintained at a certain level, indicating the beneficial effect of MAIC training on the improvement of athletes’ mindfulness levels in the short term. However, in the comparison of the post-test and continuity test, the mindfulness level of athletes does not significantly improve. The possible reason may be mainly due to the fact that several practitioners do not fully adhere to mindfulness practice during the tracking period (Rosenzweig et al., 2010). Another reason may be the game or competition itself. Therefore, the continuous effect of MAIC training on improving athletes’ mindfulness levels needs to be further explored.

From the score of the simplified flow state scale, the MAIC training intervention can effectively improve the flow state of athletes. The continuity test shows that the flow state of athletes remains at a certain level even 10 weeks after the MAIC training program intervention, indicating that MAIC training has a good effect on the continuation of the flow state level of athletes. However, in the comparison of the continuity test and post-test, the flow state of college swimmers does not significantly improve. The possible reason is that several athletes may not have continued the MAIC training. Previous literature reports a certain relationship between athletes’ mindfulness level and flow state (Hill et al., 2021). Klinger (1981) found that college basketball players who focus more on self-judgment cognition and expectation anxiety than on sports-related clues experience movement disorders, negatively affecting sports-related thinking and behavior. Enhancing mindfulness can cause subjects to not worry too much about distracting events (Klinger, 1981). The flow state experience is the best feeling of sports, which is mainly reflected in the complete concentration of attention. By comparison, MAIC training can adjust athletes’ negative emotions, calm their mood, effectively improve their attention and self-confidence, immerse them in the task of current concentration, and allow them to enter their flow state faster to improve sports performance. The results of this study are also consistent with previous literature based on MAC training, that is, a significant improvement in athletes’ sports performance (Gardner and Moore, 2004; Lutkenhouse et al., 2007). At the same time, this study expands the effect of MAIC training on the flow state experience of athletes in other types of sports.

By testing the negative emotions (anxiety and depression) and positive emotions (training and competition satisfaction) of college swimmers, the results show that the intervention of 7 weeks of MAIC training significantly reduces negative emotions and improves positive emotions. This is consistent with previous research results (Hofmann et al., 2010; Scott-Hamilton et al., 2016; Gross et al., 2018). The results of this study further support the effect of mindfulness training on negative mental states. In the MAIC theory, athletes’ awareness refers to the formation of new cognition of the meaning and values of life, a manifestation of non-persistence of thinking and contributes to the solution or improvement of current problems. Unlike the individualistic values of Western athletes, Chinese college athletes have social orientation values (such as winning glory for the country and giving priority to collective interests). This study hopes to improve the thinking flexibility of college athletes through MAIC mindfulness training to enable them to better adapt to the university’s environment and better play to their potential. After the experiment, the students were interviewed and many of them stated that they were less concerned and struggling. For example, after receiving mindfulness training, the athletes no longer stubbornly devised inconsequential reasons when the coach reprimanded them, nor wanted to vent their dissatisfaction. Rather, the athletes adopted mindfulness to let these negative internal experiences occur naturally, develop, disappear, and focus more on behaviors consistent with their values (e.g., achieving good competition results). However, after the end of the MAIC training intervention, the athletes’ negative emotions show an upward trend while the positive emotions show a decline. The reason may be that at this stage, students face the pressure of examination and competition and do not take the initiative to carry out mindfulness training. Thus, although mindfulness training has an apparent effect on the improvement of athletes’ negative and positive emotions, the effect of MAIC mindfulness training intervention gradually weakens with the passage of time. Therefore, adhering to MAIC training and forming the habit of mindfulness training after the intervention can be more beneficial to the improvement of athletes’ mental health and flow state experience. In addition, the positive psychological aspect of mental health includes training and competition satisfaction. This study found that MAIC training can improve athletes’ training and competition satisfaction. Previous literature finds that the improvement of mindfulness levels can predict the satisfaction of training competition (Blecharz et al., 2014). Mindfulness training can promote athletes’ training and competition satisfaction (Danran et al., 2020). In addition, the reduction of negative emotions may improve their flow state experience of positive emotions and sports. Whether a certain relationship exists between mindfulness and flow state experience for anxiety, depression, and training and competition satisfaction can be a focus of future research.

Finally, this study selected a sample of college student swimmers, which may differ from student-athletes in other sports. At the same time, considering the huge differences between the training and competition environment of college athletes and elite athletes, in future research, we can consider expanding the sample and increasing the scope of sports to further verify the effectiveness of the MAIC mindfulness training method. In addition, during the intervention, the athletes’ sports performance is not measured, and only the psychological state experience is examined. After the experimental intervention, the duration of the continuity test for athletes is also short at only 10 weeks, which leads to the difficulty to explain the further continuity effect of MAIC training on the athletes’ mental health and flow state. Future research can carry out an experimental design for college athletes in different sports, verify the effect of MAIC training on the “athletes” performance through competition results, and prolong the experimental period of the continuity test.

## Conclusion

The MAIC mindfulness training program based on localization design has an obvious improvement effect on college “swimmers” mindfulness level, flow state, anxiety, depression, and training competition satisfaction, with a good continuity effect. It can improve athletes’ sports experience and produce good psychological benefits. Overall, as a new mindfulness training program, MAIC provides a new way. This is the first study to explore the impact of MAIC mindfulness training on college swimmers’ flow state and mental health, which provides preliminary support for MAIC to improve the flow state and mental health of college swimmers.

## Data Availability Statement

The original contributions presented in this study are included in the article/supplementary material, further inquiries can be directed to the corresponding author.

## Ethics Statement

The studies involving human participants were reviewed and approved by the Shenyang Sport University. The patients/participants provided their written informed consent to participate in this study.

## Author Contributions

J-HN participated in the survey, data collation, and draft writing. Q-WH participated in the research guidance and manuscript editing. D-CH participated in the validation and formal analysis of the study. All authors participated in this article and approved the submitted version.

## Conflict of Interest

The authors declare that the research was conducted in the absence of any commercial or financial relationships that could be construed as a potential conflict of interest.

## Publisher’s Note

All claims expressed in this article are solely those of the authors and do not necessarily represent those of their affiliated organizations, or those of the publisher, the editors and the reviewers. Any product that may be evaluated in this article, or claim that may be made by its manufacturer, is not guaranteed or endorsed by the publisher.
